RETRACTED

# Tetra­kis(μ-2,4-difluoro­benzoato)bis­[(2,2′-bipyridine)(2,4-difluoro­benzoato)terbium(III)]

**DOI:** 10.1107/S1600536808043936

**Published:** 2009-01-08

**Authors:** Lujiang Hao, Xia Liu

**Affiliations:** a College of Food and Biological Engineering, Shandong Institute of Light Industry, Jinan 250353, People’s Republic of China; b Maize Research Institute, Shandong Academy of Agricultural Science, Jinan 250100, People’s Republic of China

## Abstract

In the centrosymmetric dinuclear title compound, [Tb_2_(C_7_H_3_F_2_O_2_)_6_(C_10_H_8_N_2_)_2_], the Tb^III^ ion is coordinated by an *N*,*N*′-bidentate 2,2′-bipyridine mol­ecule, and two *O*,*O*′-bidentate 2,4-difluoro­benzoate (dfb) anions. One of the latter also bonds to the second Tb^III^ centre through one of its O atoms. The third dfb anion bonds to one Tb atom from each of its O atoms. Thus, the three dfb species have three different coordination modes. This results in an irregular TbN_2_O_7_ coordination sphere for the metal ion. The F atoms and their associated H atoms in the simple bidentate dfb anion are disordered over two sets of sites in a 0.672 (10):0.328 (10) ratio.

## Related literature

For related literature on the biological applications of carboxyl­ates as ligands, see, for example: Serre *et al.* (2005 ▶).

## Experimental

### 

#### Crystal data

[Tb_2_(C_7_H_3_F_2_O_2_)_6_(C_10_H_8_N_2_)_2_]
*M* *_r_* = 1572.77
Triclinic,
*a* = 11.401 (1) Å
*b* = 12.189 (1) Å
*c* = 12.588 (2) Å
α = 103.99 (2)°
β = 102.90 (2)°
γ = 113.58 (2)°
*V* = 1451.5 (3) Å^3^
*Z* = 1
Mo *K*α radiation
μ = 2.52 mm^−1^
*T* = 293 (2) K
0.44 × 0.26 × 0.20 mm

#### Data collection

Bruker APEXII CCD diffractometer
Absorption correction: multi-scan (*SADABS*; Bruker, 2001 ▶) *T*_min_ = 0.403, *T*_max_ = 0.632
8233 measured reflections
5557 independent reflections
4813 reflections with *I* > 2σ(*I*)
*R*_int_ = 0.0210

#### Refinement

*R*[*F* ^2^ > 2σ(*F* ^2^)] = 0.034
*wR*(*F* ^2^) = 0.078
*S* = 1.03
5557 reflections
434 parameters
H-atom parameters constrained
Δρ_max_ = 0.60 e Å^−3^
Δρ_min_ = −0.57 e Å^−3^

### 

Data collection: *APEX2* (Bruker, 2004 ▶); cell refinement: *SAINT-Plus* (Bruker, 2001 ▶); data reduction: *SAINT-Plus*; program(s) used to solve structure: *SHELXS97* (Sheldrick, 2008 ▶); program(s) used to refine structure: *SHELXL97* (Sheldrick, 2008 ▶); molecular graphics: *SHELXTL* (Sheldrick, 2008 ▶); software used to prepare material for publication: *SHELXTL*.

## Supplementary Material

Crystal structure: contains datablocks global, I. DOI: 10.1107/S1600536808043936/hb2812sup1.cif

Structure factors: contains datablocks I. DOI: 10.1107/S1600536808043936/hb2812Isup2.hkl

Additional supplementary materials:  crystallographic information; 3D view; checkCIF report

RETRACTED

## Figures and Tables

**Table 1:** Selected bond lengths (Å)

Tb1—N1	2.565 (3)
Tb1—N2	2.586 (4)
Tb1—O6^i^	2.364 (3)
Tb1—O3^i^	2.377 (3)
Tb1—O5	2.379 (3)
Tb1—O2	2.418 (3)
Tb1—O4	2.481 (3)
Tb1—O1	2.498 (3)
Tb1—O3	2.696 (3)

Symmetry code: (i) .

## supplementary crystallographic information

### Comment

In recent years, carboxylic acids have been widely used as polydentate ligands, which can coordinate to transition or rare earth ions yielding complexes with interesting biological properties (e.g. Serre *et al.*, 2005). Herein, we report the synthesis and X-ray crystal structure analysis of the centrosymetric title compound, (I), Fig. 1.

The Tb^III^ is chelated by two 2,4-difluorobezoate anions and one 4,4'-bipyridine molecule.  Two cations are linked into dimer *via* three bridging carboxylate groups from three 2,4-difluorobezoic acid. As a result, the Tb^III^ ion is nine-coordinated with seven O atoms and two N atoms (Table 1).

### Experimental

A mixture of terbium(III) chloride (0.5 mmol), 2,4-difluorobezoic acid (1 mmol), sodium hydroxide (1 mmol), 4,4'-bipyridine (0.5 mmol), H_2_O (8 ml) and ethanol (8 ml) in a 25 ml Teflon-lined stainless steel autoclave was kept at 433 K for three days. Colourless blocks of (I) were obtained after cooling to room temperature with a yield of 16%. Anal. Calc. for C_62_H_34_F_12_Tb_2_N_4_O_12_: C 47.41, H 2.17, N 3.57%; Found: C 47.38, H 2.19, N 3.55%.

### Refinement

The H atoms were placed in calculated positions (C—H = 0.93 Å) and refined as riding with *U*_iso_(H) = 1.2*U*_eq_(C).  The F atoms of the bidenate dfb anion are disordered over two sets of sites in a 0.672 (10):0.328 (10) ratio.

### Crystal data

**Table:**

[Tb_2_(C_7_H_3_F_2_O_2_)_6_(C_10_H_8_N_2_)_2_]	*Z* = 1
*M**_r_* = 1572.77	*F*(000) = 768
Triclinic, *P*1	*D*_x_ = 1.799 Mg m^−^^3^
Hall symbol: -P 1	Mo *K*α radiation, λ = 0.71073 Å
*a* = 11.401 (1) Å	Cell parameters from 5557 reflections
*b* = 12.189 (1) Å	θ = 1.8–26.0°
*c* = 12.588 (2) Å	µ = 2.52 mm^−^^1^
α = 103.99 (2)°	*T* = 293 K
β = 102.90 (2)°	Block, colorless
γ = 113.58 (2)°	0.44 × 0.26 × 0.20 mm
*V* = 1451.5 (3) Å^3^	

### Data collection

**Table:**

Bruker APEXII CCD diffractometer	5557 independent reflections
Radiation source: fine-focus sealed tube	4813 reflections with *I* > 2σ(*I*)
graphite	*R*_int_ = 0.021
φ and ω scans	θ_max_ = 26.0°, θ_min_ = 1.8°
Absorption correction: multi-scan (*SADABS*; Bruker, 2001)	*h* = −14→13
*T*_min_ = 0.403, *T*_max_ = 0.632	*k* = −15→14
8233 measured reflections	*l* = 0→15

### Refinement

**Table:**

Refinement on *F*^2^	Primary atom site location: structure-invariant direct methods
Least-squares matrix: full	Secondary atom site location: difference Fourier map
*R*[*F*^2^ > 2σ(*F*^2^)] = 0.034	Hydrogen site location: inferred from neighbouring sites
*wR*(*F*^2^) = 0.078	H-atom parameters constrained
*S* = 1.03	*w* = 1/[σ^2^(*F*_o_^2^) + (0.0345*P*)^2^ + 0.822*P*] where *P* = (*F*_o_^2^ + 2*F*_c_^2^)/3
5557 reflections	(Δ/σ)_max_ = 0.001
434 parameters	Δρ_max_ = 0.60 e Å^−^^3^
0 restraints	Δρ_min_ = −0.57 e Å^−^^3^

RETRACTED

### Special details

**Table:**

Geometry. All e.s.d.'s (except the e.s.d. in the dihedral angle between two l.s. planes) are estimated using the full covariance matrix. The cell e.s.d.'s are taken into account individually in the estimation of e.s.d.'s in distances, angles and torsion angles; correlations between e.s.d.'s in cell parameters are only used when they are defined by crystal symmetry. An approximate (isotropic) treatment of cell e.s.d.'s is used for estimating e.s.d.'s involving l.s. planes.
Refinement. Refinement of *F*^2^ against ALL reflections. The weighted *R*-factor *wR* and goodness of fit *S* are based on *F*^2^, conventional *R*-factors *R* are based on *F*, with *F* set to zero for negative *F*^2^. The threshold expression of *F*^2^ > σ(*F*^2^) is used only for calculating *R*-factors(gt) *etc*. and is not relevant to the choice of reflections for refinement. *R*-factors based on *F*^2^ are statistically about twice as large as those based on *F*, and *R*- factors based on ALL data will be even larger.

### Fractional atomic coordinates and isotropic or equivalent isotropic displacement parameters (Å^2^)

**Table:**

	*x*	*y*	*z*	*U*_iso_*/*U*_eq_	Occ. (<1)
Tb1	0.39615 (2)	0.804496 (17)	0.439773 (18)	0.03337 (8)	
F1	0.8156 (4)	1.1600 (3)	0.2648 (3)	0.0809 (11)	
F2	0.3952 (4)	0.7245 (4)	−0.0812 (3)	0.1009 (13)	
F3	0.7957 (4)	0.9340 (4)	0.8322 (3)	0.0947 (13)	
F4	1.1389 (4)	1.1727 (5)	0.6340 (6)	0.136 (2)	
F5	−0.1318 (6)	0.5659 (8)	0.2091 (5)	0.131 (3)	0.672 (10)
F6	−0.0100 (8)	0.6768 (9)	−0.1480 (6)	0.155 (4)	0.672 (10)
F7	0.1797 (11)	0.7301 (13)	0.0303 (10)	0.100 (5)	0.328 (10)
F8	−0.3317 (10)	0.5145 (17)	0.0353 (11)	0.126 (7)	0.328 (10)
O1	0.1421 (3)	0.6937 (3)	0.3366 (3)	0.0459 (8)	
O2	0.2722 (3)	0.7141 (3)	0.2304 (3)	0.0497 (8)	
O3	0.6259 (3)	1.0197 (2)	0.5936 (3)	0.0361 (7)	
O4	0.5990 (3)	0.8317 (3)	0.5898 (3)	0.0492 (9)	
O5	0.5614 (3)	0.8920 (3)	0.3552 (3)	0.0392 (7)	
O6	0.6504 (3)	1.1034 (3)	0.3975 (3)	0.0449 (8)	
N1	0.2901 (4)	0.6091 (3)	0.4973 (4)	0.0459 (10)	
N2	0.4379 (4)	0.6128 (3)	0.3584 (3)	0.0431 (9)	
C1	0.5204 (5)	0.6201 (5)	0.2990 (5)	0.0539 (13)	
H1	0.5613	0.6955	0.2850	0.065*	
C2	0.5503 (7)	0.5218 (6)	0.2559 (5)	0.0681 (17)	
H2	0.6097	0.5311	0.2146	0.082*	
C3	0.4902 (7)	0.4132 (5)	0.2760 (5)	0.0704 (18)	
H3	0.5076	0.3455	0.2486	0.085*	
C4	0.4042 (7)	0.4023 (5)	0.3364 (5)	0.0638 (17)	
H4	0.3626	0.3270	0.3504	0.077*	
C5	0.3780 (5)	0.5031 (4)	0.3773 (4)	0.0446 (12)	
C6	0.6742 (4)	0.9489 (4)	0.6192 (4)	0.0345 (9)	
C7	0.8260 (4)	1.0066 (4)	0.6802 (4)	0.0385 (10)	
C8	0.9148 (5)	1.0685 (5)	0.6301 (5)	0.0592 (14)	
H8	0.8820	1.0786	0.5605	0.071*	
C9	1.0537 (6)	1.1153 (6)	0.6853 (7)	0.0772 (19)	
C10	1.1062 (6)	1.1066 (6)	0.7881 (8)	0.086 (2)	
H10	1.2005	1.1417	0.8242	0.103*	
C11	1.0191 (6)	1.0454 (7)	0.8389 (6)	0.0792 (19)	
H11	1.0532	1.0379	0.9095	0.095*	
C12	0.8806 (5)	0.9955 (5)	0.7837 (5)	0.0525 (13)	
C13	0.1575 (5)	0.6867 (4)	0.2397 (4)	0.0385 (10)	
C14	0.0384 (5)	0.6523 (4)	0.1333 (4)	0.0400 (10)	
C15	−0.0962 (5)	0.5956 (6)	0.1252 (5)	0.0591 (14)	
H15	−0.1166	0.5754	0.1877	0.071*	0.328 (10)
C16	−0.2018 (6)	0.5664 (7)	0.0283 (6)	0.0759 (18)	
H16	−0.2913	0.5274	0.0267	0.091*	0.672 (10)
C17	−0.1771 (6)	0.5947 (6)	−0.0640 (5)	0.0720 (18)	
H17	−0.2484	0.5771	−0.1298	0.086*	
C18	−0.0453 (7)	0.6497 (6)	−0.0581 (5)	0.0716 (17)	
H18	−0.0263	0.6684	−0.1216	0.086*	0.328 (10)
C19	0.0606 (6)	0.6780 (5)	0.0380 (5)	0.0569 (14)	
H19	0.1495	0.7160	0.0381	0.068*	0.672 (10)
C20	0.6086 (4)	0.9903 (4)	0.3307 (4)	0.0363 (10)	
C21	0.6107 (5)	0.9677 (4)	0.2092 (4)	0.0418 (11)	
C22	0.7081 (6)	1.0524 (5)	0.1800 (5)	0.0531 (13)	
C23	0.7024 (7)	1.0276 (6)	0.0660 (6)	0.0652 (16)	
H23	0.7709	1.0859	0.0489	0.078*	
C24	0.5965 (7)	0.9176 (6)	−0.0230 (5)	0.0681 (16)	
H24	0.5903	0.9012	−0.1007	0.082*	
C25	0.5015 (6)	0.8340 (6)	0.0064 (5)	0.0636 (15)	
C26	0.5055 (5)	0.8547 (5)	0.1189 (4)	0.0491 (12)	
H26	0.4385	0.7939	0.1352	0.059*	
C27	0.2154 (5)	0.6091 (5)	0.5643 (6)	0.0599 (15)	
H27	0.2191	0.6867	0.6022	0.072*	
C28	0.1331 (6)	0.5017 (6)	0.5811 (6)	0.0762 (19)	
H28	0.0830	0.5066	0.6294	0.091*	
C29	0.1267 (7)	0.3900 (6)	0.5266 (7)	0.087 (2)	
H29	0.0705	0.3154	0.5355	0.105*	
C30	0.2036 (7)	0.3854 (5)	0.4570 (6)	0.080 (2)	
H30	0.1997	0.3077	0.4189	0.095*	
C31	0.2873 (5)	0.4976 (4)	0.4440 (4)	0.0496 (13)	

RETRACTED

### Atomic displacement parameters (Å^2^)

**Table:**

	*U*^11^	*U*^22^	*U*^33^	*U*^12^	*U*^13^	*U*^23^
Tb1	0.03168 (12)	0.02483 (11)	0.04084 (14)	0.01158 (9)	0.00750 (9)	0.01636 (9)
F1	0.075 (2)	0.059 (2)	0.086 (2)	0.0040 (17)	0.046 (2)	0.0247 (18)
F2	0.109 (3)	0.095 (3)	0.055 (2)	0.024 (2)	0.030 (2)	0.000 (2)
F3	0.070 (2)	0.161 (4)	0.069 (2)	0.053 (2)	0.0260 (19)	0.071 (3)
F4	0.070 (3)	0.148 (4)	0.246 (6)	0.052 (3)	0.088 (3)	0.135 (4)
F5	0.054 (4)	0.219 (8)	0.078 (4)	0.016 (4)	0.019 (3)	0.078 (5)
F6	0.113 (6)	0.211 (9)	0.079 (5)	0.015 (5)	0.008 (4)	0.089 (5)
F7	0.051 (7)	0.170 (13)	0.094 (9)	0.037 (7)	0.027 (6)	0.104 (9)
F8	0.032 (6)	0.229 (17)	0.083 (9)	0.030 (8)	0.006 (5)	0.073 (10)
O1	0.0388 (18)	0.0500 (19)	0.0408 (19)	0.0129 (15)	0.0084 (14)	0.0241 (15)
O2	0.0381 (19)	0.057 (2)	0.0442 (19)	0.0216 (16)	0.0075 (15)	0.0124 (16)
O3	0.0339 (16)	0.0284 (14)	0.0453 (18)	0.0156 (12)	0.0066 (13)	0.0184 (13)
O4	0.0407 (18)	0.0239 (15)	0.064 (2)	0.0096 (13)	−0.0056 (16)	0.0193 (15)
O5	0.0390 (17)	0.0323 (16)	0.0500 (19)	0.0158 (13)	0.0196 (14)	0.0202 (14)
O6	0.0522 (19)	0.0304 (16)	0.051 (2)	0.0140 (14)	0.0240 (16)	0.0179 (15)
N1	0.037 (2)	0.035 (2)	0.062 (3)	0.0114 (17)	0.0091 (19)	0.0296 (19)
N2	0.042 (2)	0.0300 (19)	0.051 (2)	0.0176 (17)	0.0046 (19)	0.0161 (17)
C1	0.052 (3)	0.043 (3)	0.063 (3)	0.025 (2)	0.017 (3)	0.015 (2)
C2	0.077 (4)	0.068 (4)	0.058 (4)	0.051 (3)	0.011 (3)	0.006 (3)
C3	0.094 (5)	0.045 (3)	0.061 (4)	0.048 (3)	−0.002 (3)	0.002 (3)
C4	0.084 (4)	0.033 (3)	0.052 (3)	0.030 (3)	−0.008 (3)	0.006 (2)
C5	0.052 (3)	0.027 (2)	0.038 (3)	0.020 (2)	−0.011 (2)	0.0080 (19)
C6	0.033 (2)	0.033 (2)	0.034 (2)	0.0145 (18)	0.0048 (18)	0.0158 (18)
C7	0.034 (2)	0.032 (2)	0.048 (3)	0.0206 (19)	0.007 (2)	0.013 (2)
C8	0.050 (3)	0.054 (3)	0.084 (4)	0.026 (3)	0.025 (3)	0.041 (3)
C9	0.046 (3)	0.066 (4)	0.132 (6)	0.026 (3)	0.037 (4)	0.053 (4)
C10	0.036 (3)	0.069 (4)	0.138 (7)	0.024 (3)	0.009 (4)	0.037 (4)
C11	0.055 (4)	0.099 (5)	0.080 (4)	0.041 (4)	0.002 (3)	0.040 (4)
C12	0.042 (3)	0.067 (3)	0.050 (3)	0.030 (3)	0.009 (2)	0.024 (3)
C13	0.039 (3)	0.023 (2)	0.043 (3)	0.0114 (18)	0.005 (2)	0.0113 (19)
C14	0.038 (2)	0.036 (2)	0.035 (2)	0.013 (2)	0.0032 (19)	0.0131 (19)
C15	0.042 (3)	0.078 (4)	0.045 (3)	0.019 (3)	0.010 (2)	0.024 (3)
C16	0.040 (3)	0.103 (5)	0.059 (4)	0.025 (3)	−0.001 (3)	0.023 (4)
C17	0.057 (4)	0.076 (4)	0.052 (4)	0.027 (3)	−0.016 (3)	0.017 (3)
C18	0.080 (5)	0.075 (4)	0.043 (3)	0.025 (3)	0.009 (3)	0.028 (3)
C19	0.051 (3)	0.053 (3)	0.050 (3)	0.011 (2)	0.010 (2)	0.025 (3)
C20	0.031 (2)	0.035 (2)	0.048 (3)	0.0168 (19)	0.015 (2)	0.020 (2)
C21	0.045 (3)	0.043 (3)	0.055 (3)	0.029 (2)	0.025 (2)	0.026 (2)
C22	0.062 (3)	0.043 (3)	0.066 (4)	0.025 (3)	0.036 (3)	0.027 (3)
C23	0.092 (5)	0.068 (4)	0.082 (4)	0.052 (4)	0.063 (4)	0.048 (4)
C24	0.093 (5)	0.079 (4)	0.053 (4)	0.054 (4)	0.038 (3)	0.026 (3)
C25	0.074 (4)	0.060 (3)	0.055 (4)	0.030 (3)	0.029 (3)	0.014 (3)
C26	0.048 (3)	0.051 (3)	0.053 (3)	0.022 (2)	0.026 (2)	0.023 (2)
C27	0.051 (3)	0.054 (3)	0.089 (4)	0.024 (3)	0.028 (3)	0.047 (3)
C28	0.063 (4)	0.076 (4)	0.104 (5)	0.024 (3)	0.033 (4)	0.068 (4)
C29	0.081 (5)	0.054 (4)	0.103 (5)	0.003 (3)	0.015 (4)	0.059 (4)
C30	0.092 (5)	0.034 (3)	0.079 (4)	0.010 (3)	0.000 (4)	0.030 (3)
C31	0.052 (3)	0.028 (2)	0.050 (3)	0.011 (2)	−0.004 (2)	0.022 (2)

### Geometric parameters (Å, °)

**Table:**

Tb1—N1	2.565 (3)	C5—C31	1.463 (8)
Tb1—N2	2.586 (4)	C6—C7	1.501 (6)
Tb1—O6^i^	2.364 (3)	C7—C8	1.377 (7)
Tb1—O3^i^	2.377 (3)	C7—C12	1.377 (7)
Tb1—O5	2.379 (3)	C8—C9	1.382 (8)
Tb1—O2	2.418 (3)	C8—H8	0.9300
Tb1—O4	2.481 (3)	C9—C10	1.347 (10)
Tb1—O1	2.498 (3)	C10—C11	1.367 (10)
Tb1—O3	2.696 (3)	C10—H10	0.9300
F1—C22	1.347 (6)	C11—C12	1.373 (8)
F2—C25	1.365 (7)	C11—H11	0.9300
F3—C12	1.331 (6)	C13—C14	1.508 (6)
F4—C9	1.344 (7)	C14—C19	1.363 (7)
F5—C15	1.294 (7)	C14—C15	1.374 (7)
F5—H15	0.3691	C15—C16	1.362 (7)
F6—C18	1.353 (9)	C15—H15	0.9300
F6—H18	0.4290	C16—C17	1.346 (9)
F7—C19	1.286 (11)	C16—H16	0.9300
F7—H19	0.3654	C17—C18	1.354 (9)
F8—C16	1.392 (13)	C17—H17	0.9300
F8—H16	0.4706	C18—C19	1.362 (8)
O1—C13	1.258 (6)	C18—H18	0.9300
O2—C13	1.254 (6)	C19—H19	0.9300
O3—C6	1.259 (5)	C20—C21	1.495 (6)
O3—Tb1^i^	2.377 (3)	C21—C22	1.372 (6)
O4—C6	1.239 (5)	C21—C26	1.393 (7)
O5—C20	1.248 (5)	C22—C23	1.375 (7)
O6—C20	1.252 (5)	C23—C24	1.373 (9)
O6—Tb1^i^	2.364 (3)	C23—H23	0.9300
N1—C27	1.325 (7)	C24—C25	1.351 (8)
N1—C31	1.347 (6)	C24—H24	0.9300
N2—C1	1.315 (7)	C25—C26	1.364 (7)
N2—C5	1.345 (6)	C26—H26	0.9300
C1—C2	1.394 (7)	C27—C28	1.371 (7)
C1—H1	0.9300	C27—H27	0.9300
C2—C3	1.342 (9)	C28—C29	1.332 (10)
C2—H2	0.9300	C28—H28	0.9300
C3—C4	1.354 (9)	C29—C30	1.378 (10)
C3—H3	0.9300	C29—H29	0.9300
C4—C5	1.385 (7)	C30—C31	1.394 (7)
C4—H4	0.9300	C30—H30	0.9300
			
O6^i^—Tb1—O3^i^	75.94 (10)	C10—C9—C8	122.7 (6)
O6^i^—Tb1—O5	132.93 (10)	C9—C10—C11	119.2 (6)
O3^i^—Tb1—O5	74.31 (10)	C9—C10—H10	120.4
O6^i^—Tb1—O2	132.91 (12)	C11—C10—H10	120.4
O3^i^—Tb1—O2	78.22 (11)	C10—C11—C12	118.9 (6)
O5—Tb1—O2	74.15 (11)	C10—C11—H11	120.5
O6^i^—Tb1—O4	84.77 (12)	C12—C11—H11	120.5
O3^i^—Tb1—O4	123.24 (9)	F3—C12—C11	118.8 (5)
O5—Tb1—O4	82.03 (11)	F3—C12—C7	118.7 (4)
O2—Tb1—O4	142.07 (12)	C11—C12—C7	122.4 (6)
O6^i^—Tb1—O1	84.52 (12)	O2—C13—O1	121.4 (4)
O3^i^—Tb1—O1	81.13 (10)	O2—C13—C14	118.7 (4)
O5—Tb1—O1	125.07 (10)	O1—C13—C14	119.8 (4)
O2—Tb1—O1	52.89 (11)	O2—C13—Tb1	59.2 (2)
O4—Tb1—O1	149.70 (10)	O1—C13—Tb1	62.9 (2)
O6^i^—Tb1—N1	79.45 (12)	C14—C13—Tb1	167.8 (3)
O3^i^—Tb1—N1	145.03 (12)	C19—C14—C15	115.9 (5)
O5—Tb1—N1	139.96 (12)	C19—C14—C13	120.2 (4)
O2—Tb1—N1	101.74 (13)	C15—C14—C13	123.9 (4)
O4—Tb1—N1	78.13 (11)	F5—C15—C16	115.0 (6)
O1—Tb1—N1	72.07 (11)	F5—C15—C14	122.3 (5)
O6^i^—Tb1—N2	138.65 (12)	C16—C15—C14	122.7 (5)
O3^i^—Tb1—N2	145.39 (12)	F5—C15—H15	3.3
O5—Tb1—N2	78.18 (11)	C16—C15—H15	118.3
O2—Tb1—N2	74.34 (12)	C14—C15—H15	119.0
O4—Tb1—N2	72.15 (11)	C17—C16—C15	120.4 (6)
O1—Tb1—N2	98.32 (12)	C17—C16—F8	123.5 (7)
N1—Tb1—N2	62.76 (14)	C15—C16—F8	115.9 (7)
O6^i^—Tb1—O3	70.68 (10)	C17—C16—H16	120.1
O3^i^—Tb1—O3	73.82 (10)	C15—C16—H16	119.5
O5—Tb1—O3	66.47 (10)	F8—C16—H16	4.6
O2—Tb1—O3	136.36 (10)	C16—C17—C18	117.8 (5)
O4—Tb1—O3	49.42 (9)	C16—C17—H17	121.1
O1—Tb1—O3	148.14 (10)	C18—C17—H17	121.1
N1—Tb1—O3	120.33 (11)	C17—C18—F6	122.6 (6)
N2—Tb1—O3	113.49 (10)	C17—C18—C19	122.0 (6)
C15—F5—H15	8.4	F6—C18—C19	115.3 (7)
C18—F6—H18	8.0	C17—C18—H18	119.2
C19—F7—H19	11.1	F6—C18—H18	3.7
C16—F8—H16	9.1	C19—C18—H18	118.8
C13—O1—Tb1	90.5 (3)	F7—C19—C18	114.6 (7)
C13—O2—Tb1	94.3 (3)	F7—C19—C14	124.2 (6)
C6—O3—Tb1^i^	163.2 (3)	C18—C19—C14	121.1 (5)
C6—O3—Tb1	88.4 (2)	F7—C19—H19	4.4
Tb1^i^—O3—Tb1	106.18 (10)	C18—C19—H19	119.0
C6—O4—Tb1	99.1 (2)	C14—C19—H19	119.9
C20—O5—Tb1	136.0 (3)	O5—C20—O6	125.8 (4)
C20—O6—Tb1^i^	134.3 (3)	O5—C20—C21	115.8 (4)
C27—N1—C31	118.3 (4)	O6—C20—C21	118.4 (4)
C27—N1—Tb1	119.6 (3)	C22—C21—C26	117.6 (5)
C31—N1—Tb1	121.0 (3)	C22—C21—C20	124.3 (4)
C1—N2—C5	117.7 (4)	C26—C21—C20	118.1 (4)
C1—N2—Tb1	121.2 (3)	F1—C22—C21	119.9 (5)
C5—N2—Tb1	121.1 (3)	F1—C22—C23	118.5 (5)
N2—C1—C2	124.0 (5)	C21—C22—C23	121.5 (5)
N2—C1—H1	118.0	C24—C23—C22	120.5 (5)
C2—C1—H1	118.0	C24—C23—H23	119.7
C3—C2—C1	117.5 (6)	C22—C23—H23	119.7
C3—C2—H2	121.2	C25—C24—C23	117.6 (5)
C1—C2—H2	121.2	C25—C24—H24	121.2
C2—C3—C4	120.0 (5)	C23—C24—H24	121.2
C2—C3—H3	120.0	C24—C25—C26	123.2 (6)
C4—C3—H3	120.0	C24—C25—F2	118.2 (5)
C3—C4—C5	120.1 (5)	C26—C25—F2	118.5 (5)
C3—C4—H4	120.0	C25—C26—C21	119.4 (5)
C5—C4—H4	120.0	C25—C26—H26	120.3
N2—C5—C4	120.7 (6)	C21—C26—H26	120.3
N2—C5—C31	116.6 (4)	N1—C27—C28	124.0 (6)
C4—C5—C31	122.6 (5)	N1—C27—H27	118.0
O4—C6—O3	120.9 (4)	C28—C27—H27	118.0
O4—C6—C7	119.8 (4)	C29—C28—C27	118.4 (7)
O3—C6—C7	119.2 (4)	C29—C28—H28	120.8
O4—C6—Tb1	56.3 (2)	C27—C28—H28	120.8
O3—C6—Tb1	66.3 (2)	C28—C29—C30	119.8 (5)
C7—C6—Tb1	162.8 (3)	C28—C29—H29	120.1
C8—C7—C12	118.1 (5)	C30—C29—H29	120.1
C8—C7—C6	119.9 (4)	C29—C30—C31	119.7 (6)
C12—C7—C6	122.0 (4)	C29—C30—H30	120.2
C7—C8—C9	118.6 (5)	C31—C30—H30	120.2
C7—C8—H8	120.7	N1—C31—C30	119.9 (6)
C9—C8—H8	120.7	N1—C31—C5	116.7 (4)
F4—C9—C10	119.3 (6)	C30—C31—C5	123.4 (5)
F4—C9—C8	118.0 (6)		
			
O6^i^—Tb1—O1—C13	153.0 (3)	O1—Tb1—C6—O3	−80.4 (4)
O3^i^—Tb1—O1—C13	76.4 (2)	N1—Tb1—C6—O3	−142.7 (2)
O5—Tb1—O1—C13	12.8 (3)	N2—Tb1—C6—O3	155.0 (3)
O2—Tb1—O1—C13	−5.5 (2)	C13—Tb1—C6—O3	70.9 (7)
O4—Tb1—O1—C13	−137.2 (3)	O6^i^—Tb1—C6—C7	−178.3 (10)
N1—Tb1—O1—C13	−126.3 (3)	O3^i^—Tb1—C6—C7	−104.4 (9)
N2—Tb1—O1—C13	−68.6 (3)	O5—Tb1—C6—C7	−34.8 (9)
O3—Tb1—O1—C13	114.7 (3)	O2—Tb1—C6—C7	−22.2 (10)
C6—Tb1—O1—C13	167.7 (3)	O4—Tb1—C6—C7	82.4 (10)
O6^i^—Tb1—O2—C13	−24.4 (3)	O1—Tb1—C6—C7	166.9 (8)
O3^i^—Tb1—O2—C13	−82.2 (3)	N1—Tb1—C6—C7	104.6 (9)
O5—Tb1—O2—C13	−159.0 (3)	N2—Tb1—C6—C7	42.3 (9)
O4—Tb1—O2—C13	147.7 (2)	O3—Tb1—C6—C7	−112.7 (10)
O1—Tb1—O2—C13	5.5 (2)	C13—Tb1—C6—C7	−41.8 (13)
N1—Tb1—O2—C13	62.0 (3)	O4—C6—C7—C8	119.8 (5)
N2—Tb1—O2—C13	119.1 (3)	O3—C6—C7—C8	−56.7 (6)
O3—Tb1—O2—C13	−133.1 (2)	Tb1—C6—C7—C8	47.9 (11)
C6—Tb1—O2—C13	−171.4 (2)	O4—C6—C7—C12	−57.6 (6)
O6^i^—Tb1—O3—C6	108.2 (3)	O3—C6—C7—C12	126.0 (5)
O3^i^—Tb1—O3—C6	−171.4 (3)	Tb1—C6—C7—C12	−129.5 (9)
O5—Tb1—O3—C6	−91.8 (3)	C12—C7—C8—C9	0.5 (8)
O2—Tb1—O3—C6	−119.2 (3)	C6—C7—C8—C9	−176.9 (5)
O4—Tb1—O3—C6	8.2 (2)	C7—C8—C9—F4	178.5 (5)
O1—Tb1—O3—C6	149.0 (2)	C7—C8—C9—C10	−2.2 (10)
N1—Tb1—O3—C6	43.6 (3)	F4—C9—C10—C11	−178.5 (6)
N2—Tb1—O3—C6	−27.5 (3)	C8—C9—C10—C11	2.2 (11)
C13—Tb1—O3—C6	−158.5 (3)	C9—C10—C11—C12	−0.4 (10)
O6^i^—Tb1—O3—Tb1^i^	−80.42 (12)	C10—C11—C12—F3	178.8 (6)
O3^i^—Tb1—O3—Tb1^i^	0.0	C10—C11—C12—C7	−1.2 (10)
O5—Tb1—O3—Tb1^i^	79.59 (12)	C8—C7—C12—F3	−178.9 (5)
O2—Tb1—O3—Tb1^i^	52.25 (19)	C6—C7—C12—F3	−1.5 (7)
O4—Tb1—O3—Tb1^i^	179.60 (19)	C8—C7—C12—C11	1.1 (8)
O1—Tb1—O3—Tb1^i^	−39.5 (2)	C6—C7—C12—C11	178.6 (5)
N1—Tb1—O3—Tb1^i^	−144.96 (13)	Tb1—O2—C13—O1	−10.3 (4)
N2—Tb1—O3—Tb1^i^	143.93 (13)	Tb1—O2—C13—C14	166.2 (3)
C13—Tb1—O3—Tb1^i^	12.9 (3)	Tb1—O1—C13—O2	9.9 (4)
C6—Tb1—O3—Tb1^i^	171.4 (3)	Tb1—O1—C13—C14	−166.5 (3)
O6^i^—Tb1—O4—C6	−77.4 (3)	O6^i^—Tb1—C13—O2	161.4 (2)
O3^i^—Tb1—O4—C6	−8.0 (3)	O3^i^—Tb1—C13—O2	91.6 (3)
O5—Tb1—O4—C6	57.3 (3)	O5—Tb1—C13—O2	20.4 (3)
O2—Tb1—O4—C6	108.4 (3)	O4—Tb1—C13—O2	−70.9 (5)
O1—Tb1—O4—C6	−147.1 (3)	O1—Tb1—C13—O2	−170.2 (4)
N1—Tb1—O4—C6	−157.7 (3)	N1—Tb1—C13—O2	−120.1 (3)
N2—Tb1—O4—C6	137.4 (3)	N2—Tb1—C13—O2	−57.3 (3)
O3—Tb1—O4—C6	−8.4 (3)	O3—Tb1—C13—O2	78.8 (3)
C13—Tb1—O4—C6	151.6 (4)	C6—Tb1—C13—O2	27.0 (7)
O6^i^—Tb1—O5—C20	−43.3 (5)	O6^i^—Tb1—C13—O1	−28.4 (3)
O3^i^—Tb1—O5—C20	9.4 (4)	O3^i^—Tb1—C13—O1	−98.2 (3)
O2—Tb1—O5—C20	91.3 (4)	O5—Tb1—C13—O1	−169.4 (2)
O4—Tb1—O5—C20	−118.5 (4)	O2—Tb1—C13—O1	170.2 (4)
O1—Tb1—O5—C20	76.2 (4)	O4—Tb1—C13—O1	99.3 (4)
N1—Tb1—O5—C20	−179.2 (4)	N1—Tb1—C13—O1	50.1 (3)
N2—Tb1—O5—C20	168.2 (4)	N2—Tb1—C13—O1	112.8 (3)
O3—Tb1—O5—C20	−69.5 (4)	O3—Tb1—C13—O1	−111.0 (3)
C13—Tb1—O5—C20	82.0 (4)	C6—Tb1—C13—O1	−162.9 (5)
C6—Tb1—O5—C20	−96.6 (4)	O6^i^—Tb1—C13—C14	77.8 (17)
O6^i^—Tb1—N1—C27	18.5 (4)	O3^i^—Tb1—C13—C14	8.0 (17)
O3^i^—Tb1—N1—C27	−27.2 (5)	O5—Tb1—C13—C14	−63.2 (17)
O5—Tb1—N1—C27	167.3 (3)	O2—Tb1—C13—C14	−83.6 (17)
O2—Tb1—N1—C27	−113.4 (4)	O4—Tb1—C13—C14	−154.5 (15)
O4—Tb1—N1—C27	105.4 (4)	O1—Tb1—C13—C14	106.2 (17)
O1—Tb1—N1—C27	−69.0 (4)	N1—Tb1—C13—C14	156.3 (17)
N2—Tb1—N1—C27	−178.8 (4)	N2—Tb1—C13—C14	−140.9 (17)
O3—Tb1—N1—C27	78.6 (4)	O3—Tb1—C13—C14	−4.8 (18)
C13—Tb1—N1—C27	−90.2 (4)	C6—Tb1—C13—C14	−57 (2)
C6—Tb1—N1—C27	96.1 (4)	O2—C13—C14—C19	−14.5 (6)
O6^i^—Tb1—N1—C31	−173.7 (4)	O1—C13—C14—C19	162.0 (4)
O3^i^—Tb1—N1—C31	140.5 (3)	Tb1—C13—C14—C19	62.3 (18)
O5—Tb1—N1—C31	−24.9 (4)	O2—C13—C14—C15	166.1 (5)
O2—Tb1—N1—C31	54.3 (3)	O1—C13—C14—C15	−17.4 (7)
O4—Tb1—N1—C31	−86.9 (3)	Tb1—C13—C14—C15	−117.2 (16)
O1—Tb1—N1—C31	98.7 (3)	C19—C14—C15—F5	179.9 (7)
N2—Tb1—N1—C31	−11.0 (3)	C13—C14—C15—F5	−0.6 (10)
O3—Tb1—N1—C31	−113.6 (3)	C19—C14—C15—C16	0.1 (9)
C13—Tb1—N1—C31	77.5 (3)	C13—C14—C15—C16	179.5 (5)
C6—Tb1—N1—C31	−96.1 (3)	F5—C15—C16—C17	178.9 (7)
O6^i^—Tb1—N2—C1	−147.6 (3)	C14—C15—C16—C17	−1.2 (10)
O3^i^—Tb1—N2—C1	34.8 (4)	F5—C15—C16—F8	2.9 (13)
O5—Tb1—N2—C1	−3.0 (4)	C14—C15—C16—F8	−177.2 (10)
O2—Tb1—N2—C1	73.6 (4)	C15—C16—C17—C18	1.6 (10)
O4—Tb1—N2—C1	−88.3 (4)	F8—C16—C17—C18	177.3 (11)
O1—Tb1—N2—C1	121.2 (4)	C16—C17—C18—F6	177.0 (8)
N1—Tb1—N2—C1	−173.9 (4)	C16—C17—C18—C19	−1.0 (10)
O3—Tb1—N2—C1	−60.6 (4)	C17—C18—C19—F7	−179.9 (10)
C13—Tb1—N2—C1	96.6 (4)	F6—C18—C19—F7	1.9 (12)
C6—Tb1—N2—C1	−72.0 (4)	C17—C18—C19—C14	−0.1 (10)
O6^i^—Tb1—N2—C5	31.1 (4)	F6—C18—C19—C14	−178.3 (7)
O3^i^—Tb1—N2—C5	−146.5 (3)	C15—C14—C19—F7	−179.7 (10)
O5—Tb1—N2—C5	175.7 (3)	C13—C14—C19—F7	0.9 (12)
O2—Tb1—N2—C5	−107.7 (3)	C15—C14—C19—C18	0.6 (8)
O4—Tb1—N2—C5	90.3 (3)	C13—C14—C19—C18	−178.9 (5)
O1—Tb1—N2—C5	−60.1 (3)	Tb1—O5—C20—O6	47.9 (6)
N1—Tb1—N2—C5	4.8 (3)	Tb1—O5—C20—C21	−130.2 (4)
O3—Tb1—N2—C5	118.1 (3)	Tb1^i^—O6—C20—O5	−24.7 (7)
C13—Tb1—N2—C5	−84.8 (3)	Tb1^i^—O6—C20—C21	153.4 (3)
C6—Tb1—N2—C5	106.7 (3)	O5—C20—C21—C22	−147.8 (5)
C5—N2—C1—C2	−0.7 (7)	O6—C20—C21—C22	33.9 (7)
Tb1—N2—C1—C2	178.1 (4)	O5—C20—C21—C26	33.5 (6)
N2—C1—C2—C3	0.4 (9)	O6—C20—C21—C26	−144.8 (4)
C1—C2—C3—C4	0.0 (9)	C26—C21—C22—F1	−176.8 (5)
C2—C3—C4—C5	0.0 (9)	C20—C21—C22—F1	4.6 (7)
C1—N2—C5—C4	0.7 (7)	C26—C21—C22—C23	0.4 (8)
Tb1—N2—C5—C4	−178.1 (3)	C20—C21—C22—C23	−178.3 (5)
C1—N2—C5—C31	179.7 (4)	F1—C22—C23—C24	178.5 (5)
Tb1—N2—C5—C31	1.0 (5)	C21—C22—C23—C24	1.3 (9)
C3—C4—C5—N2	−0.4 (7)	C22—C23—C24—C25	−1.9 (9)
C3—C4—C5—C31	−179.3 (5)	C23—C24—C25—C26	0.8 (9)
Tb1—O4—C6—O3	16.1 (5)	C23—C24—C25—F2	179.6 (5)
Tb1—O4—C6—C7	−160.3 (3)	C24—C25—C26—C21	0.9 (9)
Tb1^i^—O3—C6—O4	−165.0 (7)	F2—C25—C26—C21	−178.0 (5)
Tb1—O3—C6—O4	−14.6 (4)	C22—C21—C26—C25	−1.5 (7)
Tb1^i^—O3—C6—C7	11.5 (12)	C20—C21—C26—C25	177.3 (5)
Tb1—O3—C6—C7	161.8 (4)	C31—N1—C27—C28	−1.3 (8)
Tb1^i^—O3—C6—Tb1	−150.4 (10)	Tb1—N1—C27—C28	166.8 (4)
O6^i^—Tb1—C6—O4	99.4 (3)	N1—C27—C28—C29	−0.4 (9)
O3^i^—Tb1—C6—O4	173.3 (3)	C27—C28—C29—C30	1.1 (10)
O5—Tb1—C6—O4	−117.2 (3)	C28—C29—C30—C31	−0.2 (10)
O2—Tb1—C6—O4	−104.6 (3)	C27—N1—C31—C30	2.2 (7)
O1—Tb1—C6—O4	84.5 (5)	Tb1—N1—C31—C30	−165.7 (4)
N1—Tb1—C6—O4	22.3 (3)	C27—N1—C31—C5	−175.9 (4)
N2—Tb1—C6—O4	−40.1 (3)	Tb1—N1—C31—C5	16.1 (5)
O3—Tb1—C6—O4	164.9 (5)	C29—C30—C31—N1	−1.5 (8)
C13—Tb1—C6—O4	−124.1 (6)	C29—C30—C31—C5	176.5 (5)
O6^i^—Tb1—C6—O3	−65.6 (2)	N2—C5—C31—N1	−11.0 (6)
O3^i^—Tb1—C6—O3	8.3 (3)	C4—C5—C31—N1	168.0 (4)
O5—Tb1—C6—O3	77.9 (2)	N2—C5—C31—C30	170.9 (5)
O2—Tb1—C6—O3	90.5 (3)	C4—C5—C31—C30	−10.1 (7)
O4—Tb1—C6—O3	−164.9 (5)		

Symmetry codes: (i) −*x*+1, −*y*+2, −*z*+1.
